This article has been retracted.

# Optimization of Mental Health-Related Critical Barriers in IoT-Based Teaching Methodology

**DOI:** 10.1155/2022/4602072

**Published:** 2022-04-01

**Authors:** Abhinav Juneja, Hamza Turabieh, Hemant Upadhyay, Zelalem Kiros Bitsue, Vinh Truong Hoang, Kiet Tran Trung

**Affiliations:** ^1^KIET Group of Institutions, Delhi NCR, Ghaziabad, India; ^2^Department of Information Technology, College of Computers and Information Technology, P.O. Box 11099, Taif 21944, Taif University, Saudi Arabia; ^3^BMIET, Sonepat, India; ^4^US AHO, Addis Ababa, Ethiopia; ^5^Ho Chi Minh City Open University, Ho Chi Minh City, Vietnam

## Abstract

Online learning has changed all elements of teaching of entire learning structure from primary to university level all around the world so that the challenges of online teaching are required to be optimized. The prominent objective of this manuscript is to optimize the issues of online teaching-learning in online education. Twelve issues of online teaching-learning are shortlisted by performing deep reviewing of the literature and grouping into three categories: “Students' issues,” “Common issues,” and “Teachers' issues” using the opinions of expert people. The analytical hierarchy process method is chosen for ranking of issues of online teaching. The findings can become effective in planning to get solution of the challenges of online teaching. These challenges of online teaching may lead to fragmental illness mentally over a long period of time. Because social media platforms may become an efficient tool for incorporating into online education, social media is a vital aspect of online learning. Over time, social media use may have an effect on the human brain in one way or another. The given work's exploration of online teaching-learning challenges could lead to a social media-based examination of mental illness.

## 1. Introduction

The flexible nature of online classes has proven online teaching a comprehensive element in education [1]. Online classes are a learning experience as a mode of instruction and their characteristics have met the requirements of various learners [2]. Online teaching people are supposed to have a specific set of skills [3]. Education organizations are in a prime part in enhancing the effectiveness of online learning by assisting teachers, scholars, and content refinement [4]. The union government has focused on ICT at tertiary level. For better execution of academic shift (from traditional pedagogy to online system), consequences of shift are required to be addressed [5].

Online learning is going to be instrumental for the college and university studies [6]. Considerable work has been done to check the feasibility of online classes for various parameters [7]. Several papers proposed the need of supporting academic organizations for improvement in the results of online learning [8]. Literature is deficient in case of dealing with the challenges of empowerment of online instructors and integrating techniques in methodological inquiry. Moreover, the past related work on online learning is hardly vocal about the critical optimization of competency-based teacher learning pattern [9]. Teachers build social media groups for each set of students to stream live sessions on social media platforms in order to answer questions and manage assignments. Peers might use social media platforms as an announcement board for a group of students. The use of digital content in conjunction with social media groups and channels may be beneficial. Social media is a powerful tool for aesthetically appealingly presenting a sequence of photographs or graphics.

- Therefore, it is required to address the challenges and issues of online teaching.
- Thus, the prime objectives of the current work are the exploration of challenges and issues of online teaching in Indian perspective.
- Literature survey and experts' opinions are utilized to choose challenges and issues of online teaching in Indian perspective.
- Then, AHP method is chosen to analyze the challenges and issues of online teaching in Indian perspective.
- A set of issues of online teaching-learning has been shortlisted in three categories.
- These critical challenges of online teaching from three different categories have been compared and ranked.
- The findings can become effective in planning to get solution of the challenges of online teaching.
- These challenges of online teaching may lead to fragmental illness mentally over a long period of time.
- Since social media has the potential to be an effective method for inculcating into online learning, it is an important part of online learning.
- Social media platforms are more or less addictive, and they have been linked to psychosocial problems and partial mental disease.

AHP was proposed by Saaty in 1977. This is being applied these days very frequently to compare possible options. The priorities calculated by the AHP method can be used to rank the factors. This consistency-based method is easy, robust, reliable, and mathematical.

The paper has been settled as follows: critical reviewing from concerned literature has been done in the next section. Challenges and issues of online teaching are recognized in Section 3. The proposed method has been discussed in Section 4. The calculation has been shown in Section 5. The concluding statement and scope of future work have been stated in Sections 6 and 7, respectively.

## 2. Review of Relevant Literature

Liang and Chen studied issues, potential, and challenges of online education for stakeholders while designing online activities [10]. Tai focused on the interaction in the teaching and highlighted some of the challenges and issues of online scholars as opposed to off-line scholars with the expressions of the face and gesture to further support interaction with staff [11].

Bawane and Spector reviewed the transformation learn theory [3]. Taylor explained that “competency and standards driven” work in online learning as techno-centric approach has developed one-size-fits-all concept for online teachers [12]. Valli considered online teachers who provide knowledge with theory and research for analysis and regular improvement in the level of teaching [13].

Kebritchi et al. concluded that academic organizations require to deal with the issues in online teaching and boost the efficiency of online learning [4]. Martin reviewed hundreds of articles from several online sources to much concentration on the student domain [14]. The policymakers are supposed to ensure the access of workable communication tools and better digital educational exposure and boost technology-assisted education for learners to manage and make the education structure better [5].

There are various statistical methods, which may be used for finding the relational priority of the influencing factors. The analytic hierarchy process (AHP) is an efficient method of handling the complicated decision problems when relevant data are tedious to be analyzed [15]. The AHP methodology, originally deliberated through Saaty, makes the multi-criteria decision analysis, a hierarchy for the choice [16]. AHP methodology converts the decision issue into a hierarchical model, and then, further it outlines a goal for ranking and determines various criteria and subcriteria [17]. The feature of AHP to contemplate criteria and options makes it an acceptable methodology for the industrial applications [18]. The analytic hierarchy methodology is utilized in various applications such as political science, finance, and technology [19]. AHP is beneficial for getting an optimization value with different indicators [20]. A standard objective of survey analysis, ranging from few experts to hundreds of interviewed individuals in AHP, is to gather data representative of a population, and determining the size of the sample is very crucial in this method.  Table 1 briefs few of the recent research efforts to address challenges and issues of online learning and relevant use of AHP methodology to rank the parameters.

The literature review indicates that challenges of online teaching are important from the point of view of academics, but a complicated work to be done. Thus, it is necessary to recognize issues of online teaching. Section 3 has the list and details of challenges and issues of online teaching.

## 3. Identification of Challenges and Issues of Online Teaching

Various databases (papers published in journals/presented in conferences having “Online Teaching” and “Online Classes” keywords) were reviewed, and then, twelve types of issues were categorized into three categories as per expert's opinions. The key issues include “Technical difficulties with online teaching tools,” “Over-reliance on the educator,” “Students alienation,” “LMS complications,” “Lack of real face to face interaction,” “Unstable/intermittent network connection issues,” “Data privacy/security,” “Time-consuming,” “Staying connected with passive students,” “Creating/editing/sharing online teaching content,” “Fostering an affective online learning climate,” and “Laboratory demonstration.” The identified critical barriers are categorized into three categories as “Students' issues,” “Common issues,” and “Teachers' issues.”

### 3.1. Students' Issues

Online teaching should pay special emphasis on student interaction [21]. The scholars' connection with the study management system mainly influences the student experience in case of online education [22]. Kebritchi et al. identified three types of issues in online education as issues related to teachers and students [4]. The issues related to teachers are in the four specific categories of “Technical difficulties with online teaching tools,” “Over-reliance on the educator,” “Students alienation,” and “LMS complications.”

#### 3.1.1. Technical Difficulties with Online Teaching Tools (TDWOTT)

The students lack sufficiency of time and fire of eagerness to learn newer things for online learning. The students show dissatisfaction with the technical complications installed by academic organizations for online mode, and as such, students devote much time on learning newer technologies.

#### 3.1.2. Over-Reliance on the Educator (OROE)

Most online deliveries, keeping the academic study matter in a general structure in the teaching tool, make effort to develop a comprehensive academic system that the scholars assume from course-wise and module-wise. Excessive dependency on online education becomes the issue for both instructor and learner.

#### 3.1.3. Students Alienation (SA)

Students feel very disconnected and isolated in the mode of online teaching, which influences learning. It is probably the consequence like sense of transactional gap in online mode and deficiency of communication cues (face, voice, etc.).

#### 3.1.4. LMS Complications (LMSC)

Technological complications may be because of the poor coordination of operation of the hardware and software in better online teaching.

### 3.2. Common Issues

There are few issues in online learning, which are concerned with students and teachers. The issues related to teachers are in the four specific categories of “Lack of real face to face interaction,” “Unstable/intermittent network connection issues,” “Data privacy/security,” and “Time-consuming.”

#### 3.2.1. Lack of Real Face to Face Interaction (LORF2FI)

The durable learning requires the capability for adaption to new era challenges. Effective feedback techniques are demand of hour.

#### 3.2.2. Unstable/Intermittent Network Connection Issues (UINCI)

Since online learning requires students and teachers to have access to technology, the challenges of technological accessibility cannot be ignored. Learners find the online classes as a discriminatory way by rendering them disproportionate with their mates regarding online learning technologies. Access to newer technical implications for online learning activities is hurdled by slow data speed and unstable network connectivity.

#### 3.2.3. Data Privacy/Security (DPS)

In the fast application of newer technology, educational institutes do gather huge personal info on learners and teachers and this has been creating sufficient troubling questions about data privacy.

#### 3.2.4. Time-Consuming (TC)

Even after a lot of merits related to online teaching videos, issue of long-duration videos for teaching also exists. Learners' opinion on online study material is “bulky, cumbersome, and time-consuming.” The duration of any online video is not directly proportional to the fraction of videos watched by learners.

### 3.3. Teachers' Issues

Among several ones, the pedagogical role is the most important [3]. The guide's part in the online learning needs much comprehensive as instructor work with pedagogical issues dealing with different disciplines and technologies [23]. It is notable that teachers do structure discourse of topics and dedicate huge time support for scholars in online learning [24]. The issues related to teachers are in the four specific categories of “Staying connected with passive students”; “Creating/editing/sharing an online teaching content”; “Fostering an affective online learning climate”; and “Laboratory demonstration.”

#### 3.3.1. Staying Connected with Passive Students (SCWPS)

There are different types of learners. Passive learners acquire the information but do not show interest to look for the practical applications. It is required to deliver in such a fashion that may indulge non-active students in online classes to assist to get all possible advantages.

#### 3.3.2. Creating/Editing/Sharing an Online Teaching Content (CESOTC)

Simplification of assignment is required for better understanding of learners. Teachers face issues with developing teaching matter content on LMS. Course redesign for online classes is about the technical complication of designing new teaching material and establishing favorable learning climate.

#### 3.3.3. Fostering an Affective Online Learning Climate (FAOLC)

For creating impressive online education environments, a systemized method is needed so that evaluation of the impact of education can be analyzed.

#### 3.3.4. Laboratory Demonstration (LD)

Teachers express huge emphasis on the laboratory activities for the students in online studies. Teachers demand the demonstration technologies in practice.

## 4. Methodology

To obtain the prime aim of our research work, which is the optimization of challenges of online teaching, 12 issues of online teaching are subcategorized into 2 levels (Students' issues, Common issues, Teachers' issues) as mentioned in Figure 1. The figure displays the overall ranking corresponding to complete hierarchical structure of issues taken in the current research work.

Optimization of twelve issues of online teaching is taken into three categories as Students' issues, Common issues, Teachers' issues. Analytical hierarchical process (AHA) is a hierarchy-based process; therefore, it is the best-suited multi-criteria decision-making technique for our study with a two-level categorized structure. A Web-based survey was also done with inputs from 50 individuals using Google Form to take the unbiased inputs of stakeholders to understand the priorities of the related people for various issues as potential challenges. This survey response has been duly used as a weight in the ranking of issues. Thereafter, the AHP technique has been employed in ranking these essential barriers.

### 4.1. Analytical Hierarchy Process

AHP technique calculates the consistency employing a consistency index. It permits customers to analyze the relational weight age of numerous options in context with given parameters. The analytic hierarchy process (AHP) is a math and psychology-based system for organizing and analyzing complicated decisions. The AHP has got used in many domains involving selections, during which prioritization or foretelling is required. The analytic hierarchy process (AHP) is a process that measures through pairwise comparisons and relies on expert opinion to derive priority scales. AHP permits the evaluation of comparative bias of several criteria counter to certain criteria spontaneously. It is one of the most extensively used tools for making multiple-criteria decisions. The AHP is being practiced in government policymaking, R&D, academic activities, business decisions, defense, and other many more verticals wherein decisions are made taking into account choice, preference, or prediction [25]. AHP is a versatile method for simplifying the complex MCDM issues in an organized manner by disintegrating a compound decision problem into an ordered array of relational decision members (evaluation criteria, sub-criteria, and substitutions).

The analytic hierarchy process on the basis of variable weight age methodology may adequately deal with the fixed weight ages of conventional analytic hierarchy process [26]. The analytic hierarchy process has three fundamentals such as problem decomposition, comparison judgment, and synthesis of comparative influence or ranks [27–29]. Many systems employ the AHP algorithm approach to make tough decisions. The AHP method might be considered when making decisions because data processing utilizing the AHP method will give you the greatest advice for making a big decision [30]. AHP is a versatile tool that may be used alone or in combination with other tools to solve construction decision-making issues [17, 31].

For the optimization of the challenges and issues of online teaching using the AHP approach, the identified 12 issues have been compared and evaluated using analytical hierarchical process method and further ranked in terms of priorities [32]. After identification of the hierarchical structure of AHP, further the AHP can be invoked through the following sequence of steps [33–35].

(a) Selection of criteria (*n* number of criteria).
(b) Thorough evaluation of the relational value via a sequence of pairwise associations corresponding to every decision condition employing a 9 pointer rule (1–9) to indicate their observations. The significance of values from 1 to 9 is tabulated in Table 2.
(c) Building an array of pairwise comparative square matrices (*n* × *n*) corresponding to every element in decision-making.
(d) The decision components are compared pairwise by employing *n* (*n* − 1) judgments.
(e) There is an auto-assignment of the reciprocals corresponding to every pairwise comparison.
(f) Normalization of the generated comparison matrix is performed.
(g) Hierarchical combination is obtained to generate the weights of the criteria.
(h) Eigenvalues *λ* can be calculated as the ratio of weighted sum value and criteria weight for each row of consistency matrix.
(i) Principal eigenvalue is the average of all eigenvalues. Here, we calculated the principal eigenvalue from the individual eigenvalues using the following equation:
  (1) $$\begin{array}{c} \text{Principal Eigen Value},\\ \lambda_{\max}=\sum \frac{\lambda }{n}. \end{array}$$
(j) The calculation of consistency index (AHP calculation) can be done using the following equation:
  (2) $$\begin{array}{c} \text{Consistency Index CI}=\frac{\left(\lambda_{\text{max}}-n\right)}{n-1}. \end{array}$$
(k) Random index (RI) is the value attained through arbitrarily generated pairwise comparison matrix. The significant quantum values of random index are given in Table 3.
(l) The consistency ratio (AHP calculation) is the ratio of consistency index and random index and is given as follows:
  (3) $$\begin{array}{c} \text{Consistency Ratio}\left(\text{CR}\right)=\frac{CI}{RI}. \end{array}$$

The consistency ratio must be, at most, 10% to maintain consistency in calculated judgments. A consistent ratio (CR) value of 0.1 or less is acceptable, else termed as inconsistent [17].

## 5. Results

On the basis of the data gathered by Web-based survey regarding challenges and issues of online teaching, matrices have been formulated and further calculation for calculating priorities is done by the concept of AHP. The formation of the pairwise comparison of the different categories of issues of online teaching is presented in Table 4. Table 4 has diagonal elements unity, and other elements are on the basis of survey values.

Table 4 results show that “Students' issues (0.580)” was the most important category of issues of online teaching followed by “Common issues (0.317)” and “Teachers' issues (0.110).” Further, various issues of online teaching have been ranked for each category. In Table 5, the issues under category “Students' issues” of online teaching had been checked for hierarchy.

“Technical difficulties with online teaching tools (0.606)” had been reported most important issue under category “Students' issues” of online teaching, followed by “*LMS complication* (0.220),” “Over-reliance on the educator (0.125),” and “Students alienation (0.047)” in Table 5. In Table 6, issues under category “Common issues” had been checked for hierarchy.

“Lack of real face to face interaction (0.531)” had been reported most important issue under category “Common issues” of online teaching, followed by “Unstable/intermittent network connection issues (0.338),” “Data privacy/security (0.072),” and “Time-consuming (0.047)” as shown in Table 6. The issues under category “Teachers' issues” are checked to hierarchy scale below.

Table 7 shows that “Laboratory demonstration (0.518)” had been noted as the most effective issue in category “Teachers' issues” of online teaching, followed by “Fostering an affective online learning climate (0.284),” “Staying connected with passive students (0.134),” and “Creating/editing/sharing an online teaching content (0.066).”

The consistency ratio calculated values are in the permissible range for various pairwise comparison matrices shown in Table 4 to Table 7.

We have evaluated the overall weight of every issue with the help of local weight of the issue and calculated the product by respective category's weight. After computing, overall weights of issues are tabulated in Table 8, showing that “Technical difficulties with online teaching tools,” “Lack of real face to face interaction,” and “LMS complications” are presented top three issues on the basis of overall weight age of issues.

Category ranking and overall ranking of all the issues are done in Table 8. Firstly, local weights of all twelve factors have been computed (as shown in the fifth column of Table 8), and then, the weight of their relevant category has been multiplied to get the overall weights of the factors (as shown in the sixth column of Table 8). Table 8 demonstrates that “Creating/editing/sharing an online teaching content,” “Staying connected with passive students,” and “Time-consuming issue” are presented bottom three issues based on the overall ranking of issues.

The current work has been fairly compared with the contribution from other researchers in the similar domain. Though there is no success as on date to curb the virus, some of the researchers have done wonderful efforts in uncovering challenges and issues of online teaching, which may be considered to be helpful for policymakers. The outcomes are in Table 9.

## 6. Conclusions

This study has shown a MCDM method for optimization of challenges and issues of online teaching using the AHP technique, with twelve issues (“Technical difficulties with online teaching tools,” “Over-reliance on the educator,” “Students alienation,” “LMS complications” “Lack of real face to face interaction,” “Unstable/intermittent network connection issues,” “Data privacy/security,” “Time-consuming,” “Staying connected with passive students,” “Creating/editing/sharing online teaching content,” “Fostering an affective online learning climate,” and “Laboratory demonstration”). A total of twelve critical challenges and issues of online teaching from three different categories have been compared and ranked. The current work has explored the possible issues factors, which can become a key to address the challenges of online teaching. It is obvious from the findings of the work that factors of *Students' issues*, which are influenced by factors such as “Technical difficulties with online teaching tools” and “LMS complications,” prove to be the most critical challenges of online teaching. These observations may relate the mental maladies because of social media linked with online mode of teaching and learning.

## 7. Scope for Future Work

In our study, we have applied only one technique but some other methods such as DEMATEL, TOPSIS, best-worst method, and fuzzy AHP, which can be instrumental for similar issues. Further results by applying many techniques can be compared.

## Figures and Tables

**Figure 1:** AHP-based hierarchical model to analyze issues of online teaching.

**Table 1:** Latest research of challenges and issues of online teaching.

Author	Objective and outcome
[4]	They studied about the prime issues and tactics that influence the quality of higher online education. They checked the literature that suggested to deal the challenges for online instructors
[10]	They highlighted challenges confronting online teaching
	(i) Quality assurance and standards
	(ii) Commitment versus innovation
	(iii) Copyright and intellectual property

**Table 2:** Comparison scale in AHP (Foteinopoulos et al.).

Impact of importance	Classification	Description
1	Equally significant	Two actions endorse likewise for an objective
3	Feeble significance of one over another	Familiarity and evaluation partially weigh an action to the other
5	Indispensable significant	Familiarity and evaluation strongly weigh an action to the other
7	Established significance	An action is predominantly being biased and its authority is validated
9	Complete significance	This is the maximum feasible degree of conformance
2, 4, 6, 8	Intermediary tenets	In case of a need for some negotiation

**Table 3:** RI values of *n* criteria (Saaty).

*n*	1	2	3	4	5
RI	0.00	0.00	0.58	0.90	1.12

**Table 4:** Pairwise comparison matrix of criteria.

Criteria	Students' issues	Common issues	Teachers' issues	Priority matrix	Rank
Students' issues	1	2	5	**0.580**	**1st**
Common issues	0.5	1	3	**0.317**	**2nd**
Teachers' issues	0.2	0.333	1	**0.110**	**3rd**

Maximum eigenvalue = 3.006 and C.I. = 0.003.

**Table 5:** Pairwise comparison matrix of students' issues.

Students' issues	TDWOTT	OROE	SA	LMSC	Priority matrix	Rank
TDWOTT	1	7	9	3	**0.606**	**1st**
OROE	0.142	1	4	0.500	**0.125**	**3rd**
SA	0.111	0.250	1	0.200	**0.047**	**4th**
LMSC	0.333	2	5	1	**0.220**	**2nd**

Maximum eigenvalue = 4.114 and C.I. = 0.038.

**Table 6:** Pairwise comparison matrix of common issues.

Common issues	LORF2FI	UINCI	DPS	TC	Priority matrix	Rank
LORF2FI	1	2	9	7	**0.531**	**1st**
UINCI	0.5	1	8	5	**0.338**	**2nd**
DPS	0.111	0.125	1	2	**0.072**	**3rd**
TC	0.142	0.200	0.5	1	**0.059**	**4th**

All four diagonal elements of Table 6 are unity value, and values in all other elements are on the basis of inputs. Maximum eigenvalue = 4.182 and C.I. = 0.061.

**Table 7:** Pair wise comparison matrix of teachers' issues.

Teachers' issues	SCWPS	CESOTC	FAOLC	LD	Priority matrix	Rank
SCWPS	1	2	0.5	0.25	**0.134**	**3rd**
CESOTC	0.5	1	0.2	0.142	**0.066**	**4th**
FAOLC	2	5	1	0.5	**0.284**	**2nd**
LD	4	7	2	1	**0.518**	**1st**

Maximum eigenvalue = 4.014 and C.I. = 0.00466.

**Table 8:** Computation of overall weight of issues of online teaching.

Category name	Weight of categories	Rank	Identified issues of online teaching	Local weight of issues	Overall weight of issues	Overall rank of issues
Students' issues	0.580	1st	Technical difficulties with online teaching tools (TDWOTT)	0.606	0.3514	1st
			Over-reliance on the educator (OROE)	0.125	0.0725	5th
			Students alienation (SA)	0.047	0.0273	8th
			LMS complications (LMSC)	0.220	0.1276	3rd

Common issues	0.317	2nd	Lack of real face to face interaction (LORF2FI)	0.531	0.1683	2nd
			Unstable/intermittent network connection issue (UINCI)	0.338	0.1071	4th
			Data privacy/security (DPS)	0.072	0.0228	9th
			Time-consuming (TC)	0.059	0.0187	10th

Teachers' issues	0.110	3rd	Staying connected with passive students (SCWPS)	0.134	0.0148	11th
			Creating/editing/sharing an online teaching content (CESOTC)	0.066	0.0073	12th
			Fostering an affective online learning climate (FAOLC)	0.284	0.0312	7th
			Laboratory demonstration (LD)	0.518	0.0569	6th

**Table 9:** Comparison of this study with some recent contributions.

Paper	Outcome	Present work
[5]	Their study found the challenges and issues in online teaching as the unstable network connection, intermittent signal issues, and offline conduction of classes, a lack of motivation	Our study identified the twelve key issues in online education and ranked them using MCDM technique, on the basis of a Web-based survey with inputs from fifty stakeholder individuals

[22]	They examined some of the challenges between online students and teachers. They suggested to develop flexible learning activities about course topics	Critical challenges and issues of online teaching from three different categories (Students' issues, Common issues, and Teachers' issues) have been compared by analytical hierarchy process (AHP) methodology

## Data Availability

The data will be available from the author upon request.
